The article "Green Approaches, Potentials, and Applications of Zinc Oxide Nanoparticles in Surface Coatings and Films" was published in 2022. Journal: Bioinorg Chem Appl.

# Green Approaches, Potentials, and Applications of Zinc Oxide Nanoparticles in Surface Coatings and Films

**DOI:** 10.1155/2022/3077747

**Published:** 2022-08-04

**Authors:** Rosiah Rohani, Nur Syafiqah Farhanah Dzulkharnien, Nurul Hidayah Harun, Iqma Asyila Ilias

**Affiliations:** ^1^Department of Chemical & Process Engineering, Faculty of Engineering and Built Environment, Universiti Kebangsaan Malaysia (UKM), Bangi, Selangor 43600, Malaysia; ^2^Research Centre for Sustainable Process Technology (CESPRO), Faculty of Engineering and Built Environment, Universiti Kebangsaan Malaysia (UKM), Bangi, Selangor 43600, Malaysia

## Abstract

Interest in the use of zinc oxide nanoparticles (ZnO NPs) in surface coatings and films has increased as its incorporation can significantly improve the mechanical and antimicrobial properties of coatings and film solutions. In an effort to produce green or eco-friendly products, the potential use of ZnO NPs biosynthesized from natural resources to replace conventional petroleum-derived polymers has been investigated. This review provides an insight into the growing trend of incorporating ZnO NPs into synthetic or semi-synthetic or bio-based polymeric materials via different synthesis methods as well as its characteristics and potential applications in surface coatings and films. The antimicrobial potential of ZnO NPs to inhibit the growth of various types of microorganisms as well as its use in surface coatings or films to impart antimicrobial activities that prevent the spread of microorganisms, especially the COVID-19 virus, was also discussed.

## 1. Introduction

Large structures (i.e., buildings, monuments, and ship hulls) and smaller structures (i.e., furniture, household appliances) require protection for effective long-term use. As such, surface coatings comprising polymeric materials and additives are often used to provide protection from foulants, harmful microorganisms, moisture, and UV radiation. Furthermore, in the food and beverage industry, it is crucial to use packaging film with adequate antimicrobial properties to ensure that food quality is maintained and that food is preserved from food-borne bacteria [1]. Petroleum-based polymers were previously used as coating or packaging until researchers discovered that these materials were nonbiodegradable and harmed the ecosystem [2–4]. At present, awareness on the use of eco-friendly products has risen to reduce the risk of toxicity to the environment. As such, a significant number of natural polymeric materials have been developed from plants and biological materials to provide more sustainable technologies in the future. Similarly, carbon-based and metal or metal oxide-based nanotechnologies, dendrimers, and nanocomposites are also currently being investigated as these materials have immense potential to improve the properties of films and surface coatings. Of the various metal oxide nanoparticles, zinc oxide nanoparticles (ZnO NPs) are the most commonly and widely used in various applications in the food packaging, cosmetics, biomedicine, agriculture, and coating industries as it is abundantly available in nature, low cost, biocompatible, lack pigmentation, hydrophobic, UV protective, and antimicrobial [5–8]. The addition of ZnO NPs to polymeric matrices causes surface coatings and films to develop hydrophobicity towards water due to a reduction in the hydrogen bonding within the matrices that leads to the good dispersion and less penetration of water into the surface [9]. ZnO NPs are also a potential antimicrobial agent as it is fine in size, leading to a higher interfacial area that allows the NPs to penetrate cells and, eventually, exhibit better bactericidal activity against bacteria such as *Staphylococcus aureus* (*S. aureus*) and *Escherichia coli* (*E. coli*) [10, 11].

The article "Green Approaches, Potentials, and Applications of Zinc Oxide Nanoparticles in Surface Coatings and Films" was published in 2022. Journal: Bioinorg Chem Appl.

This review is aimed at providing the current state and biosynthesis of ZnO NPs that have been incorporated into film and surface coating solutions via different methods and types of surfaces. The interactions that occur between ZnO NPs and the polymeric matrices of surface coatings and films will also be discussed. The properties of ZnO NPs were also compared with that of another NP. This review provides insight into the potential behaviour of ZnO NPs when used as an additive in surface coatings and films. This discussion elaborates each of the topics as follows:

1. Introduction
2. ZnO NPs in surface coatings and films
    2.1. Comparison of green-synthesized and nongreen-synthesized ZnO NPs
    2.2. Green approaches for surface coatings and film as biopolymeric materials
     2.2.1. Bio-based materials
     2.2.2. Plant-based materials
    2.3 Incorporation of ZnO NPs in coating materials and films and its compatibility
    2.4. Surface and coating method selection for ZnO NPs.
3. Potential of ZnO NPs in surface coating and film properties
    3.1. Mechanical properties
    3.2. Antimicrobial properties
     3.2.1. Bacteria
     3.2.2. Fungi
     3.2.3. Algae
    3.3. Antiviral potentials
    3.4. Integration of ZnO NPs with other NPs for surface coatings and films
4. Application of ZnO NPs in surface coatings and films
    4.1. Food packaging
    4.2. Textiles for biomedical applications
    4.3. Paint industry
    4.4. Marine antifouling
    4.5. Preservation works
5. Emerging research on natural polymeric materials containing ZnO NPs as a coating for antimicrobial and antiviral purposes
6. Conclusions

The article "Green Approaches, Potentials, and Applications of Zinc Oxide Nanoparticles in Surface Coatings and Films" was published in 2022. Journal: Bioinorg Chem Appl.

## 2. ZnO NPs in Surface Coatings and Films

### 2.1. Comparison of Green-Synthesized and Nongreen-Synthesized ZnO NPs

Different methods, such as direct blend with determined ZnO NPs or through top-down or bottom-up techniques, can be used to introduce ZnO NPs into surface coating and film solutions [12–14].  Figure 1 shows the two main methods of synthesizing NPs, which are the top-down or bottom-up methods. In general, the joining of multiple small particles to form a nanostructured building block of NPs is called the bottom-up approach, while a size reduction in the bulk nanomaterials is called the top-down approach. Physical and chemical methods such as laser ablation, chemical vapour deposition, ball milling, and hydrothermal as well as green methods that can be used to synthesize NP synthesis [13]. Of the physical methods, the hydrothermal method is considered the most eco-friendly and suitable for use in chemical solutions during NP synthesis.

Mohan et al. [15] described the morphological characteristics of ZnO NPs at varying temperatures and times throughout the hydrothermal method (Figure 2). They found that the synthesized ZnO NPs were spherical at 150°C after 2 hours and were in the form of nanorods at 120°C after 3 hours. Ramimoghadam et al. [25] used the hydrothermal method to synthesize ZnO with palm olein as a reducing agent. The study found that ZnO NPs were nonspherical at 120°C after 18 hours.

However, physical and chemical methods have disadvantages as they require costly equipment, high temperatures, and high pressures [10], as well as a large area to set up the machines and toxic chemicals that are hazardous to the environment. Therefore, green-synthesizing NPs is favoured over physical and chemical methods as it is an eco-friendly, feasible, safe, and cost-effective procedure that uses minimal toxic chemicals and produces less harmful by-products [13, 14].

Over the years, multiple studies have investigated green-synthesizing NPs. Agarwal et al. [26] examined green-synthesizing ZnO NPs using additives from various natural sources. This included plant extracts such as *Anisochilus carnosus*, *Plectranthus amboinicus*, *Vitex negundo*, Russian olive [27], and Rambutan peel extract [28] as well as microorganisms such as *Bacillus licheniformis, Aeromonas hydrophila,* and *Sargassum muticum* to name a few. The study reported that the presence of phytochemicals such as polyphenols in these natural strains and plant extracts acts as a reducing and capping or stabilizing agent during NP synthesis. Similarly, Obeizi et al. [29] concluded that the phytochemical constituents of *Eucalyptus globulus* essential oil act as a capping and reducing agent during ZnO NP synthesis, where the colour of the mixture was monitored from visible to light yellow.  Table 1 outlines the biosynthesis of ZnO NPs using additives from various natural sources as well as their particle sizes and morphological properties. Basnet et al. [12] successfully biosynthesized ZnO NPs using flowering plants from the *Fabaceae* and *Rutaceae* species, which is responsible for the reduction of metal salts. As the synthesized NPs were narrowly distributed, they were capable of significant antibacterial, electrochemical, sensory, and photocatalytic activity.

The article "Green Approaches, Potentials, and Applications of Zinc Oxide Nanoparticles in Surface Coatings and Films" was published in 2022. Journal: Bioinorg Chem Appl.

As seen in Table 1, chitosan, which is commonly found in animal shells, has been reportedly used to produce ZnO nanorods that could reduce aggregation and form small-sized particles (15 nm) [5]. Furthermore, plant-based oils such as palm oil comprise saturated and unsaturated fatty acids, vitamin E, tocotrienols, and vitamin A, which can be used as a bio-template to synthesize ZnO NPs owing to their mesoporous structures that promote the nucleation of ZnO NPs onto the surface of material [25]. Ramimoghadam et al. [30] used palm olein as a bio-template to synthesize ZnO NPs via the hydrothermal method. The study proposed that ZnO NPs formed due to interactions between hydroxyl (-OH) and carboxylic (-COOH) groups of fatty acids in the palm olein and the metal oxide NPs. It is believed that the carboxylic head groups combine with the surface of the nanostructure via self-assembly and later construct spherical micelles around the ZnO crystals. This inorganic-organic hybrid provides sites for the ZnO NPs to nucleate and form different morphologies [34]. Analytical instruments such as ultraviolet visible (UV-Vis) spectroscopy, Fourier transform infrared (FTIR) spectroscopy, scanning electron microscopy (SEM), and X-ray diffraction (XRD) are commonly used to determine, characterize, and compare the structure and particle sizes as well as the physical, chemical, and morphological properties of synthesized ZnO NPs. Previous studies [35, 36] reported that green-synthesized ZnO NPs with particle sizes of 30–124 nm appear as a broad and strong peak range around 350–386 nm on the UV-Vis spectra. However, chemically synthesized ZnO formed NPs with particle sizes of 18–110 nm that appear as a broad and strong peak at a similar region on the UV-Vis spectra of 350–380 nm [37, 38].  Figure 3 depicts the UV-Vis and FTIR spectra of green- and chemically synthesized ZnO NPs. As seen, peaks appear at similar wavenumber ranges, which are around 378–532 cm^−1^ and 380–667 cm^−1^, which represents the Zn-O bonds of biosynthesized and chemically synthesized ZnO NPs, respectively [17–19]. Therefore, although these ZnO NP synthesis methods vary, they both yield ZnO NPs with similar optical and physiochemical properties.

The article "Green Approaches, Potentials, and Applications of Zinc Oxide Nanoparticles in Surface Coatings and Films" was published in 2022. Journal: Bioinorg Chem Appl.

Figure 4 provides a graphical summary of the FTIR and UV-Vis spectra of nongreen- and green-synthesized ZnO NPs. The FTIR wavenumbers of ZnO NPs that had been green-synthesized using palm olein, pomelo juice, *Aegle marmelos,* and *Eucalyptus globulus* were compared with that of nongreen-synthesized ZnO NPs (hydrothermal and commercial ZnO NPs). The resulting peaks were found to range between 375 and 470 cm^−1^, indicating coherence between both green and nongreen synthesis methods. This can be attributed to the various parameters used during ZnO NP fabrication such as precursor concentration, methods, and reaction times to name a few that contribute to the shifting peaks seen in the FTIR spectra. Furthermore, some variations in wavenumber were also observed during green synthesis using different plant extracts (Figure 4). This may be attributed to the different chemical compositions of different plants, which leads to a shift in the peaks. This may also explain the wavelength seen in the UV-Vis spectra, as the ZnO NPs peaks were found to range between 360 and 380 nm.

However, XRD analysis is used to determine the crystallite state and size of the NPs using Debye Scherrer's equation as well as detect any impurities. Pavithra et al. [33] used *Citrus maxima* (Pomelo) juice as a reducing agent during ZnO NP fabrication and found that the average size of the NPs ranged between 15 and 35 nm at different concentrations. Ghasem et al. [18] successfully biosynthesized ZnO NPs using *Thymus pubescent* leaf extract and compared the XRD diffractograms of the samples with that of commercial ZnO NPs (Figure 5). The study found that the crystallite size of ZnO NPs was 58 nm, while the diffractograms were clear, indicating the high purity of the fabricated ZnO NPs. The small reduction in XRD intensity observed in the spectra may be due to the presence of plant extracts. As such, the particle sizes of ZnO NPs vary according to the plant extract that is used as a reducing agent during the synthesis process.

Table 2 shows the XRD data of ZnO NPs peaks observed in green and nongreen-synthesized ZnO NPs. As seen, the crystalline peaks of both methods were in a similar range of around 30–80° of 2*θ* with a wurtzite structure. In summary, green and nongreen-synthesized ZnO NPs exhibit similar characteristics during analysis with UV-Vis, FTIR, and XRD. As such, green synthesis should be used more frequently to fabricate NPs as it not only exhibits similar physicochemical behaviour as nongreen methods but also preserves the environment and produces fewer toxic chemicals during experimental works. The subsequent section discusses the use of green synthesis to produce NPs for surface coatings and films.

The article "Green Approaches, Potentials, and Applications of Zinc Oxide Nanoparticles in Surface Coatings and Films" was published in 2022. Journal: Bioinorg Chem Appl.

### 2.2. Green Approaches for Surface Coatings and Films as Bio-Polymeric Materials

Renewable sources such as plant-based palm olein and bio-based peptides and chitosan from chitin in crustacea exoskeletons are green and bio-organic materials that are potentially suitable for coating wood, glass, and polyurethane [39–41, 43].  Figure 6 summarizes the techniques used to fabricate biopolymeric materials for surface coatings and films.

#### 2.2.1. Bio-Based Materials

Bio-based materials such as chitosan, gelatin, and peptides contain polysaccharides that give them excellent mechanical and antimicrobial properties that are suitable for surface coating and films as well as biodegradable food packaging [42, 44]. According to Yu et al. [41], peptides can potentially be used as an antimicrobial agent on the surfaces of polyurethane catheters as it is commonly used to improve the surfaces of tools in the healthcare sector. The application is common in hospitals where catheter-associated urinary tract infections (CAUTIs) occur due to the formation of a microbial biofilm on the surface of the catheter. A coating of antimicrobial peptides was found to inhibit the development of both Gram-negative (gr−) and Gram-positive (gr+) microbial bacteria on the surface by up to 99.9%. This provides some insight into the efficacy of functionalizing surfaces with peptide biomaterials to inhibit bacteria and biofilm formation.

#### 2.2.2. Plant-Based Materials

Plant-based materials such as starch are preferred as food packaging film due to their homogeneous matrices [45]. However, in recent times, plant oils such as acylated palm olein (APO), acylated jatropha oil (AEJO), and acrylated epoxidized palm oil (AEPO) have been used and modified to exhibit high yield and better performance, such as UV-curable and high-hardness surface coatings [46].  Figure 7 depicts the chemical structures and condition of modified jatropha oil and acrylated epoxidized palm oil.

These materials are more suited for use as a UV-curable surface coating than unmodified or epoxidized oil due to their unique fatty acid composition and high percentage of cross-links (Table 3). Highly viscous materials are preferable as they prevent unnecessary spreading and indicate high fluid concentration. The mechanical properties of acylated oils such as APO and AEJO indicate significant durability as a coating material on wood and mil steel coating, respectively. Furthermore, these green materials could also provide good adhesion on surfaces post-UV treatment coating and are suitable to replace current petroleum-based coatings.

The article "Green Approaches, Potentials, and Applications of Zinc Oxide Nanoparticles in Surface Coatings and Films" was published in 2022. Journal: Bioinorg Chem Appl.

Although plant-based polymers are less scratch-resistant than petroleum-based coatings, different initiators or resins can be added to these plant- or bio-based materials to improve their scratch resistance. Al-Naamani et al. [47] investigated the antifouling activity of synthesized chitosan-ZnO NPs coating by adding acetic acid into the solution. The study found that the chitosan-ZnO nanocomposite hybrid coating had the lowest bacterial concentration after four weeks under light conditions, indicating excellent antifouling activity. Marsi and Rus [48] combined palm oil with titanium dioxide (TiO_2_) at different metal oxide percentages to improve the surface coating properties. It is noteworthy that the incorporation of metal oxides could enhance the properties of bio-sources and eventually be used as an alternative to nonbiodegradable polymers.

### 2.3. Incorporation of ZnO NPs in Coating Materials and Films and Its Compatibility

ZnO NPs are commonly integrated with synthetic, semi-synthetic, and biopolymeric materials via blending and have been used as a finishing on various surfaces. As seen in Figure 8, resins and polymeric materials successfully merged with ZnO NPs.

However, a few factors such as the pH, concentration, size, smoothness, and distribution of the NPs need to be taken into consideration when selecting coating materials and films to be embedded with ZnO NPs. This is because the inhomogeneity of ZnO NPs in a matrix, due to a high concentration of NPs, could cause agglomeration that degrades its performance and aesthetical values [49, 50]. Aung et al. [19] fabricated a *Jatropha curcas* oil-based polyol comprising polyurethane (PU) and different concentrations of ZnO NPs that possess anticorrosive properties. The study found that low concentrations (<7%) of ZnO NPs facilitated smooth dispersion while agglomeration started to occur at ZnO NPs concentrations exceeding 7%, which decreased the anticorrosive performance of the coating.  Figure 9 depicts the opacity of steel surfaces coated with different concentrations of ZnO NPs-AEJO. As seen, ZnO NPs-AEJO with the highest concentration of fillers provided the clearest opacity on steel surfaces. This indicates that suitable concentrations of NPs that can be used in the coating industry to maintain the surface aesthetical values, colour, or opacity of the biopolymer itself.

Weththimuni et al. [20] incorporated a bio-based resin made of shellac insects with ZnO NPs that had been functionalized with a silane compound to increase the compatibility between the inorganic NPs and the organic shellac. The study found that the particle size of functionalized ZnO NPs was smaller than that of pristine ZnO NPs due to the presence of silane, which was used to reduce NP aggregation. Therefore, functionalizing the ZnO NPs could minimize agglomeration as well as enhance the properties of the materials. Furthermore, fabricating nanocomposites by combining ZnO NPs and polymers such as tetramethylolpropane triacrylate (TMPTA) and 2-hydroxy-2-methylpropiophenone (Darocur 1173) linked with chitosan also exhibited good compatibility at sufficient compositions [19].

The article "Green Approaches, Potentials, and Applications of Zinc Oxide Nanoparticles in Surface Coatings and Films" was published in 2022. Journal: Bioinorg Chem Appl.

Shaban et al. [21] investigated the hydrophobicity of ZnO NPs in a synthetic monoethanolamine (MEA) stabilizer. The study found that hydrophobicity increased as the ZnO NPs concentration increased before it dropped at 0.7 M. At a low ZnO NPs concentration (0.1 M), the hydrophobicity was low as the surface was not completely coated and less hydrogen bonding. A ZnO NP concentration of 0.5 M was found to provide optimum coating due to the presence of more oxygen vacancies and active sites for adhesion on the surface. The ZnO NPs were found to agglomerate and become less uniform at concentrations exceeding 0.5 M, which reduces their ability to resist the penetration of water. Therefore, the concentration of ZnO NPs used in coatings and films is another vital factor that needs to be taken into account, to prevent agglomerations that reduce its performance.

The dispersion of ZnO NPs in a surface coating can also be affected by its pH. This is because NPs tend to agglomerate and nucleate at low pH due to the presence of fewer hydroxyl groups (OH^−^) in the solution [51]. Therefore, it is advisable to maintain a pH of 7 as this could facilitate the homogeneous distribution of the ZnO NPs.

The morphological properties of ZnO NP coatings such as homogeneity, dispersion, size, and shape can be elucidated through scanning electron microscope (SEM) and transmission electron microscope (TEM) images. Amjadi et al. [42] observed the SEM images of ZnO NP-chitosan and found that the small ZnO NP particulates (23–62 nm) were able to enter the porous structure of the chitosan nanofibers (CHNF) (25–64 nm). Furthermore, ZnO NPs can also fill the spaces in the gelatin matrix by increasing cross-linking to yield a stronger structure against water [52, 53]. Afsharpour et al. [10] fabricated uniformly dispersed ZnO NPs that had been functionalized with Klucel™ G hydroxypropyl cellulose and observed its morphological behaviour. The study discovered that the integration of ZnO NPs into the structure of the fiber cellulosic material yielded better mechanical properties, relative to that of pristine ZnO NPs. Therefore, ZnO NPs could prevent the leaching of excessive Zn^2+^ ions as well as improve the stability and ability of polymeric matrices to adhere to surfaces and films [19, 31]. ZnO NPs have shown potential to be encapsulated with various materials to obtain nano-sized particles that could promote better stability and antimicrobial properties, and reduce leaching of Zn^2+^ ions [54, 55], relative to exposure to UV [56].

The article "Green Approaches, Potentials, and Applications of Zinc Oxide Nanoparticles in Surface Coatings and Films" was published in 2022. Journal: Bioinorg Chem Appl.

According to the Food and Drug Administration (FDA), macrosized ZnO is safe for use in the eco-friendly food packaging industry [57, 58]. However, there are still concerns over the use of nano-sized ZnO as it has the tendency to release excessive Zn^2+^ ions, especially for applications in the food industry and marine environments [59]. This is because excessive Zn^2+^ ions could cause cytotoxicity in aquatic organisms, which will eventually lead to toxicity in humans. Furthermore, certain solvents such as water can promote the leaching of ions. The following equation explains the possible ionization of Zn^2+^ ions from ZnO NPs after exposure to water [47]:

(1) $$\begin{array}{c} \text{ZnO}+{\text{H}}_{2}\text{O}⟶{\text{Zn}}^{2+}+2{\text{OH}}^{-}. \end{array}$$

The leaching and aggregation of Zn^2+^ ions during the production of ZnO NPs has become a major concern. As such, researchers have discovered a way of overcoming this issue by encapsulating ZnO NPs in a polymeric agent, which modifies its antimicrobial activity. Therefore, the addition of a support matrix to ZnO NPs is an alternative that could be used to overcome the toxicity issue [60]. Tissera et al. [56] used poly (acrylonitrile) (PAN) nanofibers to encapsulate ZnO NPs for better photocatalytic activity. They found out that the ZnO NPs with an average size of 35 nm had successfully embedded in the PAN nanofibers through SEM photomicrographs.

Tajau et al. [14, 46] reported the synthesis of nano-sized particles of acrylated palm olein (APO) NPs using gamma radiation techniques for use as an encapsulating agent to deliver the drug, paclitaxel, to combat cancer cells. The fine size of the APO NPs is believed to be able to trap ZnO precursors and, eventually, generate stable ZnO NPs [24, 62, 63]. Furthermore, encapsulation is thought to counteract the toxic risks to humans, animals, and the environment as it can reduce the amount of ZnO NPs leakage, which consequently decreases the release of Zn^2+^ from coating solutions.

### 2.4. Surface and Coating Method Selection for ZnO NP Fabrication

As the dispersion of ZnO NPs in a biopolymer increases the transparency of the biopolymer film, it is suitable for surface coatings as it will not change the aesthetics, which can damage the value of the surface. Furthermore, as the polymer is found to be less in water in the presence of ZnO NPs, it makes coated surfaces such as steel, glass, and wood become more durable [9]. Films commonly used as food wrappings also need to maintain their quality to ensure that the packaged food can last longer [64]. Coatings and films that contain ZnO NPs possess excellent antimicrobial, anticorrosive, UV protective, and mechanical properties in addition to super-hydrophobicity.  Figure 10 depicts several coating techniques that integrate ZnO NPs into polymeric matrices.

The article "Green Approaches, Potentials, and Applications of Zinc Oxide Nanoparticles in Surface Coatings and Films" was published in 2022. Journal: Bioinorg Chem Appl.

In the roller coating method, bar rollers automatically apply a uniform thickness of the coating solution on a flat surface. Aung et al. [19] used the roller coating method to coat steel, while Mizielińska et al. [65] used a similar method to coat polyethylene film via the use of UV radiation. This technique is preferable as it can be conducted at room temperature under a medium-pressured UV lamp [66]. However, it may not be suitable for coating nonflat surfaces due to its uneven outer layer. In such instances, spray-based techniques are preferred, especially for nonflat materials such as 3D helical springs and furniture as well as surfaces with low mechanical and thermal resistance such as paper [67]. Spray-based coating is done by manually or automatically spraying a certain amount of liquid coating solution onto the surface of a material using special equipment such as a spray gun [68]. Some spray guns require gas (i.e., nitrogen) and suitable pressure for operation.

In the textile industry, the dip-spin coating method is commonly used to coat the surfaces of fiber-textured materials as it provides strong adhesion to ensure that the ZnO NPs are embedded on each strand. Meanwhile, smaller fabrics are immersed in a selected coating solution, withdrawn, and then dried at a suitable temperature. This process is repeated in cycles to ensure that the surfaces are well-coated. Altering parameters such as the type and concentration of the coating solution could modify the ability of NPs to adhere to the surface of a textile. Rădulescu et al. [31] altered coating solutions by varying the volume of ZnO NPs in a mixture of orange oil and sodium hydroxide (NaOH). Apart from textiles, this method can also be used to coat wood samples. Additionally, the adhesion quality of the NPs to the surfaces of a material can be improved by merging the dip-coating technique with other methods, such as precipitation and hydrothermal [22].

Sol-gel spin coating is another technique that is commonly used to coat cotton with ZnO NPs [21]. This is done by dropping a coating solution on the surface of a sample and then spinning the sample with the help of vacuum suction at a constant rate and time, to ensure the stability of the sample during coating. The coated sample is then dried to remove excess coating solvent. This technique is more advantageous and reliable than dip coating due to its easy thickness control, better homogeneity, and suitability for large-sized textiles such as clothing fabrics [62].  Figure 11 illustrates the dip-spin coating method on a material that comprises fibrous structures to ensure that each strand of the fiber is well-coated.

The article "Green Approaches, Potentials, and Applications of Zinc Oxide Nanoparticles in Surface Coatings and Films" was published in 2022. Journal: Bioinorg Chem Appl.

The brushing method is commonly used to coat surfaces such as buildings with NPs. This is a feasible method of depositing polymeric resins containing ZnO NPs on surface [24]. Weththimuni et al. [61] used the brushing technique to coat maple wood with a shellac-based varnish embedded with ZnO NPs to reduce the occurrence of photo-and biodegradation as well as impart antifungal properties. The number of brushings was fixed to 20, and the brush was adjusted to be perpendicular to the brushed area for uniformity during the experiment. The number of coatings was found to affect the performance of the ZnO NPs in the coating solution. Exceeding a certain number of coats was found to cause the ZnO NPs to agglomerate, which was unfavourable for the structure [21]. Lastly, the casting method is frequently used in the fabrication of ZnO NPs that are integrated with bio-composite films such as gelatin, starch, and chitosan [9, 35, 42]. In this method, ZnO NPs are first sonicated to form a homogeneous solution before it is poured into a moulder such as Petri dish or polystyrene plate and left to dry. The presence of ZnO NPs in the film enhanced the potent mechanical properties of these biopolymeric films specifically.

## 3. Potential of ZnO NPs in Surface Coating and Film Properties

### 3.1. Mechanical Properties

Mechanical properties are the physical properties that a material exhibits upon the application of forces. Variations in materials, techniques, and parameters could change the mechanical properties of materials. Therefore, the presence of ZnO NPs on the surface of a coating or film will modify and improve its mechanical characteristics such as hardness, ability to adhere to surfaces, and UV resistance, as well as its tensile characteristics such as elongation time to break (ETB), ultimate tensile strength (UTS), and Young's Modulus (YM).  Table 4 provides a list of the mechanical properties of surface coatings and films with and without the use of ZnO NPs.

As seen in Table 4, NPs can improve the physical properties of natural-based polymers such as chitosan, gelatin, and starch. For instance, the presence of ZnO nanofillers in reinforcing starch film was found to enhance its barrier and thermal stability performance [63]. These improvements in mechanical properties are mainly due to good interaction between the NPs and the matrix as well as the homogeneous dispersion of the NPs in the matrices [69]. Chang et al. [70] suggested that the high value of Young's modulus for starch-ZnO NPs system was due to the strong molecular interaction between ZnO NPs and starch chain. However, this metal oxide-loaded matrix was less water soluble due to the formation of hydrogen bonds between the ZnO NPs and the starch, which decreased the OH^−^ group in the matrix. Furthermore, the starch-ZnO NPs matrix became more hydrophobic, relative to the original starch, due to the presence of ZnO NPs that filled up the empty spaces and consequently facilitated hydrogen bonding [71]. Amjadi et al. [42] reported that ZnO NPs with gelatin-based film had low water solubility, indicating the strong water resistance of the film. These physical properties may be due to the ability of ZnO NPs to fill gaps in the film matrix, which reduces the mobility of its chains resulting in higher cross-linking and better water resistance [53]. Das et al. [72] also suggested that the water resistance of a synthesized bio-composite consisting of chitosan loaded with ZnO NPs was due to the formation of a three-dimensional (3D) network of NPs that provides a stabilization effect to the chitosan.

The article "Green Approaches, Potentials, and Applications of Zinc Oxide Nanoparticles in Surface Coatings and Films" was published in 2022. Journal: Bioinorg Chem Appl.

Furthermore, hardness is also an important mechanical property that is commonly tested. This test is performed by firmly pushing the lead of a pencil into the surface of a material at a 45° angle. The hardness of a surface that had been coated with a coating containing ZnO NP filler was found to have increase as a 6H pencil was required to scratch the coated surface, while a HB pencil was sufficient to scratch the uncoated surface [73, 74].

### 3.2. Antimicrobial Properties

ZnO NPs are known to possess antimicrobial properties that can inhibit the presence of microorganisms such as fungi and bacteria. According to extant studies [1, 5, 8, 16, 21, 29, 36, 75], ZnO NPs of various shapes, of spherical, nanorods, cubic hexagonal or irregular, and various sizes (<200 nm) have been found to exhibit potential antimicrobial properties.  Figure 12 provides a list of the bacteria and fungi that have been successfully inhibited by ZnO NP materials.

The agar diffusion method is commonly used to test the antimicrobial activity of a compound. A broth solution is first prepared using a specific agar media depending on the microorganisms tested. In general, yeast extract glucose chloramphenicol (YGC) agar is used for fungi, while nutrient agar is used for bacteria [8, 29]. The broth solution is then incubated and plated until it solidifies. A broth containing a specific concentration of the selected microorganisms is then swabbed onto the solidified agar media before NPs are deposited on the agar. Antimicrobial potential is then determined by measuring the inhibition zone (Figure 13) or optical density (OD) to observe microorganism concentrations [8, 21].

The article "Green Approaches, Potentials, and Applications of Zinc Oxide Nanoparticles in Surface Coatings and Films" was published in 2022. Journal: Bioinorg Chem Appl.

Another method that can be used to determine antimicrobial activity is microbroth dilution [42]. In this technique, microorganisms are first prepared according to McFarland No. 1 opacity in sterile normal saline. A series of broths containing different ZnO NP dilutions are then prepared before the microorganism suspension is added. The solutions are incubated after which the bacterial growth in the well is observed via minimum inhibition concentration (MIC) [76].

Some of the several proposed mechanisms by which ZnO NPs inhibit microorganisms include the ionization of ZnO NPs, the photocatalytic activity of the reactive oxygen species (ROS) produced by the ZnO NPs, and the accumulation of ZnO.  Figure 14 depicts a simplified schematic of the possible mechanism that ZnO NPs use to kill microorganisms.

ZnO NPs are believed to undergo ionization, which releases Zn^2+^ ions that disturbs the cell wall of a microorganism. These Zn^2+^ ions eventually pass through the cells and disrupt the enzymatic system of the cell, which subsequently kills the microorganisms [77–79]. The idea has been supported by Kanmani and Rhim [80] in which they explained that the presence of the metal may form pits in the cell membrane permeability, leading to cell death. Another proposed mechanism of ZnO NPs in inhibiting the bactericidal strain is through the generation of ROS [81, 82]. Jin et al. [83] described that ZnO NPs and their aggregates can produce ROS including singlet oxygen (^1^O_2_), hydroxyl radicals (^.^OH), hydrogen peroxide (H_2_O_2_), and superoxide (O^−•^) under UV irradiation. They initiated oxidative stress of mitochondria and endoplasmic reticulum dysfunction in *E. coli* resulting in irreversible membrane damage, DNA mutation, and death in *E. coli*. According to their study, the antibacterial potential of ZnO NPs was not mediated by Zn^2+^ ions, which suggested that the Zn^2+^ ions were not escaped from NP or NP network. Hübner and Haase explained that zinc itself is redox-inactive and always present in the valence state Zn (II) in biological systems causing the zinc unable to directly participate in redox reactions [84]. Lastly, an accumulation of ZnO NPs on the cell wall of a bacteria due to electrostatic forces causes the internalization of ZnO NPs that hinder the metabolism of the cell and cause its destruction [85, 86]. This suggested mechanism is more efficient under UV radiation as the UV light provides better conductivity that can activate interactions between the ZnO NPs and the cell wall of the microorganism [87].

The article "Green Approaches, Potentials, and Applications of Zinc Oxide Nanoparticles in Surface Coatings and Films" was published in 2022. Journal: Bioinorg Chem Appl.

#### 3.2.1. Bacteria

ZnO NPs possess antimicrobial properties towards various species of gr− bacteria such as *E. coli*, *Pseudomonas aeruginosa* (*P. aeruginosa*), *Xanthomonas oryzae pv. oryzae (Xoo) strain GZ 0003*, *Pseudoalteromonas nigrifaciens*, *Klebsiella pneumoniae* (*K. pneumoniae*), and *Pseudomonas fluorescens* [1, 16, 21, 36, 42, 47] and gr+ bacteria such as *S. aureus*, *Bacillus subtilis* (*B. subtilis*), and *Listeria monocytogenes* [1, 21, 42]. However, ZnO NPs have lower antibacterial activity towards Gram-positive bacteria as they have thicker cell walls unlike Gram-negative bacteria, which have a thinner outer membrane composed of lipopolysaccharide and peptidoglycan that is less of a barrier to ROS [88]. Therefore, gr− bacteria are more sensitive to antibacterial activity than gr+ bacteria [36, 42].

The antimicrobial activity of the synthesized ZnO NPs is usually determined using common antibiotics such as Chloramphenicol, Ampicillin, and Gentamycin, to study the effectiveness of materials in these properties. According to previous studies [21, 31], materials coated with ZnO NPs exhibit good antimicrobial activity against *S. aureus* and *K. pneumoniae* but are less effective against *E. coli, Salmonella typhimurium,* and *B. subtilis* than commercially available antibiotics. Therefore, coating materials loaded with ZnO NPs can inhibit the growth of bacteria over a period of time.

#### 3.2.2. Fungi

Apart from bacteria, ZnO NPs also show significant antimicrobial activity against fungi species such as *Candida albicans* (*C. albicans*, white mould) and *Aspergillus Niger* (*A. niger*, black mould) [29, 36]. Afsharpour and Imani [8] found that ZnO NPs successfully inhibit the growth of white mould and black mould on the surface of paper. As such, coatings containing ZnO NPs have been used on varnished wood surfaces and exhibit excellent antifungal characteristics that inhibit growth of undesired fungi on the surface of the wood [20].  Figure 15 displays the photographs of the surface of wood (a) with plain varnish and (b) coated with ZnO NPs. As seen, fungal (mould) was clearly present on wood coated with non-ZnO NPs varnish, while wood coated with ZnO NPs was clear. This proved that ZnO NPs had the potential to treat surfaces infected by fungi. However, Anupama et al. [36] found that the antimicrobial activity of ZnO NPs against fungi species, *A. Niger* (black mould) and *Fusarium solani*, was almost negligible, which contradicts the former statement. These results may vary from one another due to the synthesis methods, the type of fungus, and the size of the NPs used.

The article "Green Approaches, Potentials, and Applications of Zinc Oxide Nanoparticles in Surface Coatings and Films" was published in 2022. Journal: Bioinorg Chem Appl.

#### 3.2.3. Algae

Other than bacteria and fungi, ZnO NPs can also inhibit the growth of algae species. The interactions between NPs and algae are similar to its interactions with bacteria, in which it generates ROS, accumulates ZnO NPs or Zn^2+^ ions in cells, and disrupts the cell membrane with electrostatic forces [89]. According to Abiraman et al. [5], coatings containing ZnO NPs were 75–90% effective at inhibiting the growth of marine algae strains such as *Chlorella*, *Amphora*, and *Arthrospira* that were deposited on the antifouling paint and left for 30 days in sea and freshwater. Al-Naamani et al. [47] synthesized a ZnO coating to act as an antidiatom agent for *Navicula* sp and found that coatings with ZnO NPs particle sizes ranging between 50 and 60 nm possess good antidiatom activity. Apart from antimicrobial potential, ZnO NPs are also reported to have the ability to act as antiviral agents.

### 3.3. Antiviral Potentials

Viruses such as influenza A, H1N1, human papilloma virus (HPV), and severe acute respiratory syndrome coronavirus 2 (SARS-CoV-2) can be transferred from one host to another via aerosolized particles and droplets on surfaces [90]. Therefore, it is imperative that alternatives to prevent such viruses from spreading in the community be found. One way of combatting the spread of such viruses is by creating coatings with antiviral potential. Silver nanoparticles (Ag NPs) are well-known antiviral agents that have been commercialized by the paint industry. However, the antiviral potential of ZnO NPs has yet to be fully explored and warrants more extensive study. To date, only in situ experiments involving virus-infected cells and computational chemistry studies have been used to study the antiviral potential of ZnO NPs. According to these studies, two mechanisms correspond to NPs and viruses: (i) a reduction in the replication of RNA viruses via the penetration of ZnO NPs or Zn^2+^ ions into virus cells and (ii) the formation of free radicals from ZnO NPs [91]. Recent studies by Ghaffari et al. [92] have concluded that ZnO NPs substantially inhibit H1N1 and SARS-CoV-2 by 52.2% and 45%, respectively. An in vivo study has also been conducted to determine the efficacy of using ZnO NPs to clear planar warts on 16 patients with a median age of 29 years over four weeks. The study found a significant reduction in the diameter, surface area, and volume of the warts beginning from week two [93], indicating that spherical ZnO NPs ranging between 20 and 50 nm in size are effective at inhibiting plantar warts caused by HPV. However, as the study was only conducted over a four-week period, a longer study is necessary to obtain more reliable results.

The article "Green Approaches, Potentials, and Applications of Zinc Oxide Nanoparticles in Surface Coatings and Films" was published in 2022. Journal: Bioinorg Chem Appl.

El-Megharbel et al. [37] used ZnO NPs ranging between 40 and 60 nm in size as an antiviral agent for SARS-CoV-2 [94]. The study found that nanocomposite materials comprising ZnO NPs and polyethylene glycol (PEG) possess good antiviral characteristics and cytotoxicity towards the virus [95]. Adhikari et al. [22] developed an anti-SARS-CoV-2 face mask that employed ZnO nanoflower NPs on a cotton surface. The study conducted a simulation that showed the mechanism by which the ZnO NPs inhibited the growth of SARS-CoV-2 by trapping, denaturing, and removing its spike proteins. The bacteria, *P. aeruginosa*, was used for the antimicrobial test as the amino acids present in *P. aeruginosa* are very similar to the spike receptor-binding domain (RBD) of SARS-CoV-2.

### 3.4. Integration of ZnO NPs with Other NPs for Surface Coatings and Films

ZnO NPs possess better mechanical strength and antimicrobial potential than other NPs such as Ag NPs and TiO_2_ NPs. As such, ZnO NPs have been added to surface coatings and films that contain other NPs to overcome the weakness of pristine NPs. For instance, Ag NPs are highly toxic to human cells and the environment as it releases Ag^+^ ions. Therefore, Nguyen et al. [75] immobilized Ag NPs on ZnO NPs to overcome the toxicity issue and impart better antimicrobial characteristics. Lallo da Silva [11] integrated ZnO NPs with TiO_2_ NPs as ZnO NPs are biocompatible and have better photocatalytic activity, higher durability, and higher heat resistance than TiO_2_ NPs alone. Peighambardoust et al. [35] examined and compared the mechanical properties of starch films containing different types of metallic NPs. The study concluded that starches with ZnO NPs had higher elastic break (EB) and YM than starches with Ag NPs and copper oxide nanoparticles (CuO NPs). The study also observed that agglomeration did not occur between NPs and starch due to increased surface contact between the NPs and their matrix [2]. A similar result was also found by Amjadi et al. [42].

The integration of two or more antimicrobial NPs, by combining with ZnO NPs in a system, fosters bio-activity against infections and controls resistance of bacterial or fungal strains. For instance, the addition of different percentages of magnesium (Mg) dopants in ZnO NPs coatings on cotton has been found to vary the performance of ZnO NPs [21]. Increasing the Mg doping percentage was found to decrease the hydrophobicity of the surface coating as the Mg deteriorates the crystallinity of the coating structure. Furthermore, hybrid metallic NPs has been found to exhibit better performance in terms of mechanical strength, antimicrobial activity, and toxicity. As such, this method could be used to reduce the use of expensive materials such Ag NPs, in either coatings or materials. Moreover, Ag NPs and ZnO NPs could be combined to reduce the material cost while retaining their antimicrobial properties.

The article "Green Approaches, Potentials, and Applications of Zinc Oxide Nanoparticles in Surface Coatings and Films" was published in 2022. Journal: Bioinorg Chem Appl.

## 4. Application of ZnO NPs in Surface Coatings and Films

Coating a material is an important part of ensuring that its performance, and aesthetics do not degrade easily [5]. In recent times, ZnO NPs have garnered considerable attention among researchers and industries for use in various applications such as food packaging film, biomedical textiles, and the paint industry due to its outstanding mechanical and antimicrobial activities [22].  Figure 16 provides a list of applications related to ZnO NPs surface coatings and films.

### 4.1. Food Packaging

Although the FDA has deemed macrosized ZnO safe, ZnO NPs are highly toxic to humans and are a major concern that requires alternatives to overcome the toxicity issue [96]. However, emerging ZnO NPs with polymeric materials or other NPs could reduce or eliminate its toxicity. To that end, gelatin and starch are biomaterials that are commonly used to promote green food packaging films over petroleum-based films [35, 42]. Embedding ZnO NPs in the gelatin matrix of food packaging film has been found to provide better mechanical strength as well as protect food for a long time. The incorporation of ZnO NPs in gelatin films has been found to successfully inhibit the growth of food-borne bacteria, such as *P. aeruginosa, S. aureus*, and *E. coli*. Meanwhile, chitosan NPs loaded with ZnO NPs have also been used as food packaging to reduce the release of excessive Zn^2+^ ions into food. Fruits and vegetables such as oranges, apples, carrots, and broccoli are commonly required good food packaging to prevent the growth of bacteria and mould that could deteriorate the freshness of these foods. According to previous literature [9], the food (carrot) was preserved for five days due to effective interactions between the ZnO NPs and the hydroxyl (-OH) and amino (-NH_2_) groups in the chitosan as well as the presence of the bio-active components of azadirachtin in the neem oil.

Apart from food packaging, ZnO NPs are also useful in the textile industry, especially for biomedical applications, as they could potentially control antimicrobial activities and protect the surface of textiles from microorganisms. The application and functionality of ZnO NPs in the textile industry is discussed in the next subtopic.

The article "Green Approaches, Potentials, and Applications of Zinc Oxide Nanoparticles in Surface Coatings and Films" was published in 2022. Journal: Bioinorg Chem Appl.

### 4.2. Textiles for Biomedical Applications

The use of ZnO NPs in the textile industry is increasing due to its unique properties such as hydrophobicity, UV protection, self-cleaning, and antimicrobial activity [49], which could prevent the transmission and spread of harmful microbials. The advantages of ZnO NP coatings in the textiles industry have contributed to its wider application such as medical equipment, home curtains, beddings, and car seats to name a few. For instance, face masks and personal protection equipment (PPE) will perform better with these coatings as they provide an extra barrier for microbial organisms to overcome. Furthermore, cotton and wound dressings coated with ZnO NPs exhibit significant antimicrobial activity against *E. coli* [21, 22, 31]. Furthermore, reducing or killing bacteria on these textiles may reduce odour as well as help them last longer by preventing the formation of mould.

Cotton is generally used in daily life due to its softness and affinity to skin [97, 98]. As cotton fabrics comprise threaded textures that are rich in OH^−^ groups, they are easily stained by liquids that eventually lead to bacterial growth. Recently, ZnO NPs have been reported to create superhydrophobic surfaces on cotton fabrics via the *Lotus* effect [99, 100]. Wound dressings have also been innovated by adopting nanotechnologies such as the addition of NPs, including ZnO NPs, that could improve their antimicrobial activity [31]. The antiviral potential of ZnO NPs can be used to make cotton-based face masks, especially to prevent SARS-CoV-2 infection [22]. This is an important discovery as face masks are one of the new norms implemented to prevent SARS-CoV-2 from spreading.  Figure 17 presents the mechanisms by which face masks coated with ZnO NPs interact with SARS-CoV-2. As seen, the virus is expected to bind to the ZnO nanoflowers on the surface of the cotton face mask, leading to the denaturation of its spike proteins and its eventual death. The benefits of using ZnO NPs in the paint industry are discussed in the next subtopic.

### 4.3. Paint Industry

Furniture, decorations, and walls are familiar surfaces in homes that could harbor and support the growth of microorganisms such as fungi, viruses, and bacteria, especially in moist environments. Wood such as maple and rubber wood are popular choices of materials for furniture and decorations in homes. However, they are easily exposed to the formation of fungi and bacteria. Therefore, the addition of ZnO NPs into resin coatings such as varnish could improve the quality of wood surfaces as ZnO NPs are less pigmented, hydrophobic, and self-cleaning, which is favoured in painting applications as the coating needs to be transparent, restrict moisture penetration as well as require only a few cleanings [20]. Paints containing ZnO NPs have been found to possess effective antifungal, antimicrobial, anticorrosive, antidiatom, and self-cleaning properties [23]. However, the current antimicrobial coatings available in the industry contain a non-natural chemical that may be harmful to the environment. Therefore, green alternatives that use plants and bio-based materials for coatings can overcome this issue as well as the shortage of nonrenewable resources such as petroleum.  Figure 18 shows that a few items that use commercial paints such as PU, enamel, and acrylic, with ZnO NPs, perform better as coatings [101]. Furthermore, ZnO NPs are also compatible with resins due to their good blending ability as well as their ability to maintain its viscosity and consistency. As wood is commonly used in the marine industry to construct boats and jetties, paints that contain ZnO NPs have good antimicrobial properties that can be used to support antifouling activity. This will be elaborated upon in the next subtopic.

The article "Green Approaches, Potentials, and Applications of Zinc Oxide Nanoparticles in Surface Coatings and Films" was published in 2022. Journal: Bioinorg Chem Appl.

### 4.4. Marine Antifouling

Antifouling agents are important in the marine industry as the presence of foulants such as marine algae and bacteria can degrade mechanics and aesthetics of infrastructure. For instance, an increase in the growth of microorganisms on the hull of ships can contribute to decreased vessel performance such as slower speed and higher fuel consumption [102, 103]. The major concern about antifouling coatings is the release of toxic biocides that contain harmful compounds such as lead, arsenic, and mercury [104, 105]. Despite the ability of these compounds to prevent fouling activities, their drawbacks should not be overlooked. As such, other options such as zwitterionic silane and poly (ethylene glycol) nanofibrous mesh should be investigated. However, these materials are expensive and less eco-friendly. To that end, Abiraman et al. [5] introduced a chitosan-ZnO nanocomposite coating that offers marine-friendly antifouling activity. Another application of ZnO NPs in surface coatings is preservation, which will be discussed in the subsequent subtopic.

### 4.5. Preservation Works

The preservation of old manuscripts and buildings are necessary to restore culture heritage sites. As such, ZnO NPs are widely used in the preservation industry due to their resistance to microorganisms and its self-cleaning ability [106–109]. As seen in Figures 19(a) and 19(b), a ZnO NPs coating can be used to maintain the aesthetics of an old manuscript. Furthermore, the antimicrobial properties of these NPs can protect the surface of the paper from destructive microorganisms such as *C. albicans* (white mould), fungus, and dirt as well as provide a UV protective barrier. Protective coatings such as paper varnish could also be blended with ZnO NPs to preserve coloured oil paintings in museums for a longer period of time [110]. Additionally, ZnO NPs are also used as reinforcing fillers in steel surface coatings as it is cheap, convenient, biocompatible, anticorrosive, antibacterial, and antifungal as well as possesses good mechanical properties and is nontoxic [111–113]. Moreover, the addition of consolidates or water-repellent materials blended with ZnO NPs can reduce the formation of *A. niger* (black mould) on stone monuments by tenfold [24]. As seen in Figures 19(c) and 19(d), varnishes containing ZnO NPs (C1 and C2) improved the properties of the surface in terms of mould formation and colour compared to uncoated surfaces (A1 and A2) and varnishes without ZnO NPs (B1 and B2) after 40 days. Therefore, ZnO NPs are suitable for use in the preservation of old manuscripts and buildings.

The article "Green Approaches, Potentials, and Applications of Zinc Oxide Nanoparticles in Surface Coatings and Films" was published in 2022. Journal: Bioinorg Chem Appl.

## 5. Emerging Research on Natural Polymeric Materials Containing ZnO NPs as a Coating for Antimicrobial and Antiviral Purposes

At present, the paint industry has extensively explored the integration of nanotechnology to maintain the conditions and properties of material surfaces. Therefore, utilizing ZnO NPs in surface coatings and films has greatly contributed to various applications such as paint, textiles, and food packaging, to name a few. The incorporation of ZnO NPs in biopolymeric materials via green approaches has attracted significant attention among researchers in the hope of sustaining the environment. Therefore, future studies may use natural materials to synthesize ZnO nanocomposite coatings without removing the natural synthesizing agent. For instance, palm olein (PO), a natural polymer, has been found to be able to synthesize ZnO NPs as NPs are amorphous and possess potential biodegradable chemical compositions [46]. As PO is usually used in cooking and will be removed after several uses as waste cooking oil (WCO), instead of throwing the WCO away, it can be recycled and converted into a useful product such as biodiesel, thereby preventing pollution. Furthermore, PO can be converted to APO, whose derivatives could potentially be used as a surface coating for wood. However, one of the major concerns of using natural polymers is the poor mechanical strength of most biopolymer coatings as they are not compatible with synthetic coatings [114, 115]. Therefore, the use of additional of NPs, including ZnO NPs, is expected to mitigate the issue.

The article "Green Approaches, Potentials, and Applications of Zinc Oxide Nanoparticles in Surface Coatings and Films" was published in 2022. Journal: Bioinorg Chem Appl.

Parameters such as material type, method of use, temperature, and reaction time should be taken into consideration to control the adhesion performance and quality of ZnO NPs. The use of polymeric nanomaterials with stable encapsulating properties and biocompatibility is favoured to maintain the features and values of ZnO NPs. As most natural-based biopolymers contain −H groups that facilitate surface modifications that improve the properties of nanocomposites, it birthed the idea of using green materials to encapsulate ZnO NPs so that these eco-friendly materials have the potential to prevent the SARS-CoV-2 virus [116]. Nevertheless, material cost, safety, skills, and setup for in vitro studies are some of the challenges that warrant serious consideration to avoid accidents during experimentation.

## 6. Conclusion

In conclusion, ZnO NPs hold great potential as surface coatings and films due to their ability to blend with polymeric solutions. Apart from excellent antimicrobial activity against bacteria, fungi, algae, and viruses, ZnO NPs are also highly durable in external conditions such as UV, friction, and humidity, which is vital for coating and film applications. The addition of ZnO NPs in polymer matrices seems to be an effective way of overcoming issues such as agglomeration and Zn^2+^ ion leaching. It is strongly recommended that future studies examine assimilating bio-sources or waste into ZnO NPs and coating and film solutions to support green technologies. As most of the biopolymeric materials available for surface coatings and films have inadequate mechanical properties to replace nonsustainable materials, ZnO NPs are an excellent filler that can enhance this physical behaviour. It is hoped that this review spurs the exploration of ZnO NPs in coating materials and films, especially natural-based, so that more emerging research on sustainable bio-composites will be published.

## Figures and Tables

**Figure 1:** Two main approaches in synthesizing NPs.

**Figure 2:** Fabrication of ZnO NPs using the hydrothermal method. Adapted from Ref. [15].

**Figure 3:** FTIR spectra of (a) green-synthesized and (b) nongreen-synthesized ZnO NPs. Spectra were taken from Refs. [16, 17].

**Figure 4:** Summary of (a) wavenumber from FTIR and (b) wavelength from UV-Vis spectra of nongreen- and green-synthesized ZnO NPs from previous literatures.

**Figure 5:** XRD spectrum of green-synthesized ZnO NPs (green synthesized-GS) and commercialized ZnO NPs (commercial-C). The image was adopted from Ref. [18].

**Figure 6:** Two sources for biopolymeric materials from animal parts or plant extract.

The article "Green Approaches, Potentials, and Applications of Zinc Oxide Nanoparticles in Surface Coatings and Films" was published in 2022. Journal: Bioinorg Chem Appl.

**Figure 7:** The chemical structure of acrylated epoxidized palm oil (AEPO) for wood surface coating and acrylated epoxidized jatropha oil (AEJO) for wood and mild steel surface coating. Adapted with permission from Ref. [19]. Copyright 2020 American chemical society.

**Figure 8:** List of polymeric materials mixed with ZnO NPs.

**Figure 9:** Steel surfaces coated with acrylated epoxy jatropha oil incorporated with ZnO NPs at different concentrations. Adapted with permission from Ref. [19]. Copyright 2020 American chemical society.

**Figure 10:** Coating techniques to deposit ZnO NPs coatings on different materials as found in literature studies. Techniques: casting, roller coating, spray-based, brushing on surfaces such as wood, cement slab, paper, and steel.

**Figure 11:** Illustration of the techniques used to coat NPs on textiles; (a) dip-coating and (b) spin coating.

**Figure 12:** Antimicrobial properties of ZnO NPs against different types of microorganisms.

**Figure 13:** Measuring the inhibition zone of samples against methicillin-resistant staphylococcus aureus bacteria.

**Figure 14:** Simplified diagram showing the mechanisms of antimicrobial activity of ZnO NPs through (1) formation of zinc (Zn2+) ions produced by the NPs, (2) reactive oxygen species (ROS) of OH− ions, O_2_^−^ ions or H2O2, (3) accumulation of small-size ZnO NPs in the cell.

**Figure 15:** Comparison of fungal growth after 40 days on wood (a) coated with plain varnish and (b) wood coated with varnish containing ZnO NPs. The photogram was adopted from Ref. [20].

**Figure 16:** Applications of ZnO NPs coatings and films.

**Figure 17:** (a) ZnO NPs coating on cotton to form an antiviral filter for face masks, (b) SEM images of ZnO nanoflowers coated on cotton fabric and (c) water droplets fully absorbed on the untreated cotton surface and (d) water droplet with high contact angle on ZnO NP-coated cotton surface indicating good hydrophobicity. Reprinted with permission from Refs. [21, 22]. Copyright (2021) American chemical society.

**Figure 18:** Different surfaces coated with paint containing ZnO NPs. (a) Carbon steel surface coated with paint blended with 2% ZnO NPs, (b) clear PU and white PU blended with ZnO NPs for wood and cement slab panels, respectively, (c) and (d) display common wood used in households. The image was taken from Ref. [23].

**Figure 19:** Conditions of old manuscript (a) before and (b) after coating with ZnO NPs, (c) building for the in situ experimentation of coating, and (d) the tested area results between coated and uncoated parts. Illustration was taken from Ref. [24].

**Table 1:** Biological materials used for ZnO NP synthesis via different synthesis methods.

Green materials	Size of NPs (nm)	Shape of ZnO NPs	Method of synthesis	Zinc precursor	Ref
Chitosan	15 (width) and 110	Nanorods	Chemical conversion	Zinc sulfate pentahydrate	[5]
Essential oil of eucalyptus globulus	40	Irregular needle and spherical	Biosynthesis	Zinc acetate dihydrate	[29]
Chamomile flower, olive leave, and red tomato	49.8–191.0 40.5–124.0 65.6–133.0	Pure crystalline or cubic	Biosynthesis	Zinc oxide	[16]
Palm olein	20–500	Nanoflower	Hydrothermal	Zinc acetate	[30]
Orange oil	20	Hexagonal and polyhedral	Precipitation	Zinc nitrate	[31]
*V. arctostaphylos* L.(Caucasian whortleberry)	12	Nearly spherical	Microwave-assisted green synthesis	Zinc nitrate	[32]
*Citrus maxima* (pomelo) juice	10–20	Nearly spherical	Solution combustion	Zinc nitrate	[33]

The article "Green Approaches, Potentials, and Applications of Zinc Oxide Nanoparticles in Surface Coatings and Films" was published in 2022. Journal: Bioinorg Chem Appl.

**Table 2:** The comparison for spectroscopy data between nongreen-synthesized and green-synthesized ZnO NPs.

Green or non-green	Method/source of ZnO NPs	XRD (ZnO crystal analysis)	Ref
Nongreen	Ion exchange with zeolite	Crystalline peaks at 2*θ* = 4°–70° range of sharp intensity. The structure found is hexagonal wurtzite.	[1]
	Hydrothermal	Crystalline peaks at 2*θ* = 31.52°, 34.15°, 35.95°, 47.28°, 56.28°, 62.52°, 66.11°, 67.68°, 68.83°, 72.22°, and 76.84°. Hexagonal structure with different crystal planes, (100), (002), (101), (102), (110), (103), (112), and (201).	[37]
	Commercial (Systerm Chempur)	Crystalline peaks at 2*θ* = 31.98°, 34.63°, 36.46°, 47.69°, and 56.73°. Corresponds to hexagonal wurtzite structure.	[39]
	Commercial (NanoSany, Iran)	Crystalline peaks at 2*θ* = 30°–80° range of sharp intensity. Size of NPs = 58 nm.	[40]
Green	Synthesized with essential oil of eucalyptus globulus	Crystalline peaks at 2*θ* = 31.74°, 34.38°, 36.21°, 47.49°, 56.54°, 62.86°, 66.43°, 67.89°, 68.99°, 72.76°, and 76.94°. Hexagonal structure with different crystal planes, (100), (002), (101), (102), (110), (103), (200), (112), (201), (004), and (202) with lattice constants a = b = 3.2578 Å, c = 5.2179 Å. Size of NPs = 24 nm.	[12, 41]
	Synthesized with palm olein	Crystalline peaks at 2*θ* = 30°–70° range. Hexagonal wurtzite structure with different crystal planes, (100), (002), (101), (102), (110), (103), (200), (112), (201). Referred to standard value of JCPDS No. 36-1451.	[32]
	Synthesized with citrus maxima (Pomelo) juice	Crystalline peaks at 2*θ* = 30°–80° range. Hexagonal wurtzite structure with different crystal planes, (100), (002), (101), (102), (110), (103), (200), (112), (201), (004), (202). Referred to standard value of JCPDS No. 36-1451. Crystalline size: 15–35 nm.	[35]
	Synthesized with Aegle marmelos	Crystalline peaks at 2*θ* = 30°–80° range with high and sharp intensities. Hexagonal wurtzite structure with crystal planes (100), (002), and (101) of lattice constants *a* = *b* = 3.2417 Å, *c* = 5.1876 Å. Size of crystals: 20 nm	[17]

The article "Green Approaches, Potentials, and Applications of Zinc Oxide Nanoparticles in Surface Coatings and Films" was published in 2022. Journal: Bioinorg Chem Appl.

**Table 3:** Comparison between nonderived and derived plant-based materials.

Sample	Colour	Viscosity	OOC	IV	AV
PO	Yellow	72.00	0.05	60.98	0.03
EPO	Light yellow	117.0	3.20	9.49	1.55
AEPO	Dark brown	497.5	0.88	25.50	48.25

**Table 4:** List of mechanical data for coatings/films embedded with ZnO NPs.

Coating/film materials	Substrate	Mechanical data		Water activity		Ref.
		Coating/film materials only	Coating/film materials with ZnO NPs	Coating/film materials only	Coating/film materials with ZnO NPs	
Jatropha oil-based epoxy acrylate (AEJO)	Steel	Adhesion: 45.7 psi Pencil hardness: HB Scratch hardness: 1.0°N	Adhesion: 133.0 psi Pencil hardness: 6 H Scratch hardness: 2.4 N	WCA: 85.1°	WCA: 99.35°	[8]

Hydroxypropyl cellulose (HPC)	Paper	TS in machine direction: 42.75 N TS in cross direction: 17.76 N	TS in machine direction: 44.48°N TS in cross direction: 19.20 N	—		[9]

Monoethanolamine (MEA)	Cotton fabric	ZnO-coated surface test details UV illumination: 700 minute Outdoor exposure time: 40 days Scratch resistance test: 1500-mesh sandpaper with 1 kg load at 1 cm/s speed for 20 cycles. Conclusion, ZnO coating still gives hydrophobicity property to surface after all these tests.		WCA: 0° (No coating)	WCA: 154°	[35]

Gelatin	Film	ETB: 18.98% UTS: 6.015 MPa YM: 142.85 MPa	ETB: 12.70% UTS: 18.29 MPa YM: 853.76 MPa	Moisture absorption percentage of bare gelatin is reduced with the addition of ZnO nps to 5.57%		[38]

Starch (st)	Film	ETB: 98.00% TS: 3.67 MPa YM: 7.80 MPa	ETB: 55.67% TS: 7.5 MPa YM: 25.44 MPa	%solubility: 32.25% WVP (10^−7^ g/mhPa): 11.46	%solubility: 24.07% WVP (10^−7^ g/mhPa): 8.32	[19]

Chitosan	Film	—		% solubility in water: 78.3%	% solubility in water: 43.2%	[42]

Tensile strength (TS), elongation to break (ETB), ultimate tensile strength (UTS), Young's modulus (YM), water contact angle (WCA), water vapour permeability (WVP), and percentage of solubility in water (% solubility).

## Data Availability

No data were used to support this study.
